The article "New Psychoactive Substances: Evolution in the Exchange of Information and Innovative Legal Responses in the European Union" was published in 2020. Journal: Int J Environ Res Public Health.

# New Psychoactive Substances: Evolution in the Exchange of Information and Innovative Legal Responses in the European Union

**DOI:** 10.3390/ijerph17228704

**Published:** 2020-11-23

**Authors:** Maria Rosaria Varì, Giulio Mannocchi, Roberta Tittarelli, Laura Leondina Campanozzi, Giulio Nittari, Alessandro Feola, Federica Umani Ronchi, Giovanna Ricci

**Affiliations:** 1 National Center on Addiction and Doping, Istituto Superiore di Sanità, Viale Regina Elena 299, 00161 Rome, Italy; mariarosaria.vari@iss.it; 2 International School of Advanced Studies (ISAS), University of Camerino, Piazza Cavour 19/f, 62032 Camerino, Italy; 3 Department of Anatomical, Histological, Forensic and Orthopedic Sciences, Sapienza University of Rome, Viale Regina Elena 336, 00161 Rome, Italy; roberta.tittarelli@uniroma1.it (R.T.); federica.umanironchi@uniroma1.it (F.U.R.); 4 Research Unit of Bioethics and Humanities, Campus Bio-Medico University of Rome, Via Alvaro del Portillo 21, 00128 Rome, Italy; l.campanozzi@unicampus.it; 5 School of Pharmacy and Health Products, Telemedicine and Telepharmacy Center, University of Camerino, Via Madonna Delle Carceri 9, 62032 Camerino, Italy; giulio.nittari@unicam.it; 6 Department of Experimental Medicine, University of Campania “Luigi Vanvitelli”, Via Luciano Armanni 5, 80138 Naples, Italy; alessandro.feola@icloud.com; 7 Medico Legal Section, School of Law, University of Camerino, Piazza Cavour 19/f, 62032 Camerino, Italy; giovanna.ricci@unicam.it

**Keywords:** new psychoactive substances, early warning system, European drug legislation

## Abstract

At the end of 2019, the European Monitoring Centre for Drugs and Drug Addiction was monitoring around 790 new psychoactive substances, more than twice the total number of controlled substances under the United Nations Conventions. These substances, which are not subject to international drug controls, include a wide range of molecules, including the assortment of drugs such as synthetic cannabinoids, stimulants, opiates, and benzodiazepines. Most of them are sold as “legal” substitutes for illicit drugs, while others are intended for small groups willing to experiment with them in order to know their possible new effects. At the national level, various measures have been taken to control new substances and many European countries have responded with specific legislation in favor of consumer safety and by extending or adapting existing drug laws to incorporate the new psychoactive substances. Moreover, since 1997, an early warning system has been created in Europe for identifying and responding quickly to the risks of new psychoactive substances. In order to establish a quicker and more effective system to address the criminal activities associated with new dangerous psychoactive substances, the European legal framework has considerably changed over the years.

The article "New Psychoactive Substances: Evolution in the Exchange of Information and Innovative Legal Responses in the European Union" was published in 2020. Journal: Int J Environ Res Public Health.

## 1. Introduction

New psychoactive substances (NPS) are “substances of abuse, either in a pure form or a preparation, that are not controlled by the 1961 Single Convention on Narcotic Drugs or the 1971 Convention on Psychotropic Substances, but which may pose a public health threat” (Article 1 of Council Framework Decision 2004/757/JHA of 25 October 2004, as amended by Directive (EU) 2017/2103 of the European Parliament and of the Council of 15 November 2017) [1]. The NPS market comprises numerous substances, such as stimulants, synthetic cannabinoids, benzodiazepines, opioids, hallucinogens, and dissociatives. NPS represent a major challenge in the international scenario of drug users. Since the early 2000s, NPS have been limited to a handful of substances and not scheduled or listed under the drug control conventions. Therefore, these substances have started being sold in the open market, as their sale has not been expressly prohibited by international regulation. The globalization combined to web technologies has contributed to the development of the NPS market. Since 2015, approximately 400 previously reported NPS are detected every year [2]. At the end of 2019, the European Monitoring Centre for Drugs and Drug Addiction (EMCDDA) was monitoring around 790 NPS, 53 of which were reported for the first time in Europe in 2019 [2,3,4,5,6,7,8,9]. During 2018, European law enforcement agencies reported close to 64,800 NPS seizures to the EU Early Warning System (EWS) [2]. Of these, approximately 40,200 seizures were reported by EU member states [2]. Most of the seizures concerned more than 5.6 tons of new synthetic psychoactive substances, mostly in the form of powders [2]. A total of 4212 L of liquids and 1.6 million tablets and capsules containing NPS were also found [2]. However, since 2015, this trend seems to have stabilized or slowly declined. This emergence has led to a modification of traditional approaches of drug monitoring, surveillance, control, and public health responses over the years. In 1997 (European Council, 1997), a system was implemented in Europe for identifying, exchanging information, and responding quickly to the risks of NPS [10,11]. This system is based on a three-step legal framework of early warning, risk assessment, and fast-track control measures (political decision at the European level enacted through national legislations) [12,13,14]. The EMCDDA is responsible for the first two steps in this system. However, this strategy had to evolve to keep pace with the NPS trends, and in the 2005 Framework Decision (Council of the European Union, 2005), the complete mechanism was established. In 2011, the European Commission communicated its will to produce stronger EU level regulations in this area (European Commission, 2011a), and in 2013, new proposals for regulation and directives on the treatment of NPS in Europe were presented (European Commission, 2013). In April 2014, the European Parliament indicated its strong support for these proposals, but discussions among EU member states were stalled over the correct legal basis for the proposals. In April 2016, these discussions were resolved, and the proposals were once again put forward on August 29 with a slightly amended legal basis. New legislation was introduced in November 2018, which retained the European three-step approach, but considerably strengthened the existing procedures thanks to a single risk assessment report on the potential risks posed by several NPS with a similar chemical structure. Shorter deadlines also applied to these new procedures. Under the latest legislation, other EU agencies have been involved, including the European Centre for Disease Prevention and Control (ECDC), the European Chemicals Agency (ECHA), and the European Food Safety Authority (EFSA). The manuscript aims to retrace, over the years, the legal framework and aspirations of the European Union at both the national and the international level with the purpose of rapid identification, assessment, and response to the health and social dangers posed by the NPS.

The article "New Psychoactive Substances: Evolution in the Exchange of Information and Innovative Legal Responses in the European Union" was published in 2020. Journal: Int J Environ Res Public Health.

## 2. Materials and Methods

A comprehensive literature search was performed on European institutional websites (EUR-Lex, Publications Office of the European Union, EMCDDA, European Council of the European Union, Gazzetta Ufficiale Italiana, United Nations Office on Drugs and Crime (UNODC)) to describe the European legislation related to the evolution of the information exchange network on new synthetic drugs in Europe. The following research terms were used: information on new synthetic drugs, NPS Legal Response, EMCDDA, EU EWS. Search was done in English and Italian languages and all the documents were independently screened and selected by three of the authors to assess their relevance for the aim of the review. The 8000 sources found were screened to exclude the sources and papers not suitable for the purpose of the review. Only 16 documents (7 in the website of the EMCDDA, 1 in the website of the UNODC, 5 in the site of EUR-lex, 3 in the site of the Publications Office of the European Union, and 1 in the website of the European Council of the European Union) were included in this work. Only the publications that were considered relevant by at least two of the manuscript authors were selected.

The article "New Psychoactive Substances: Evolution in the Exchange of Information and Innovative Legal Responses in the European Union" was published in 2020. Journal: Int J Environ Res Public Health.

## 3. Results

### 3.1. Evolution and Legal Responses to the Markets of New Psychoactive Substances

In order to counter this phenomenon, since 1997, the EMCDDA and the European Union Agency for Law Enforcement Cooperation (Europol) with the support of the EU member states, the European Medicines Agency (EMA), and the European Commission have been playing an important role in assessing the risks connected to the spread of NPS by collecting information on their diffusion in the European markets and monitoring the signals of threats to the national and global public health security agencies [15]. The first legislations (1997 and 2005) allowed the partners to develop a sophisticated EWS to follow NPS, as well as a structure that would allow, to date, scientific risk assessments.

### 3.2. Exchange of Information on New Synthetic Drugs (1997)

Joint Action 96/699/JHA, Article K.3 of the Treaty on EU, has been intended to establish for the first time a more cohesive mechanism for the transmission and diffusion of the results of drug profiling in the EU. It has provided the exchange of information regarding the chemical profiling of the most common illicit drugs and other psychotropic substances. The Europol Drugs Unit (EDU) was appointed to produce and send the information format to all the member states. In 1997, a system for rapid exchange of information on NPS and risk assessment was implemented so that the control measures for psychotropic substances enforced in the member states could also be applied to them (97/396/JHA) [16]. The Joint Action concerned NPS which, although not currently listed in the Schedules of Psychotropic Substances of the 1971 United Nations Convention, showed limited therapeutic effect and constituted a threat to public health similar to that of the substances listed in Schedules I and II of that Convention. The action concerned end products and not precursors, for which Community arrangements were provided for under Council Regulation (European Economic Community—EEC) No. 3677/90 of 13 December 1990. Specific measures were taken to discourage the diversion of substances to the illicit manufacture of narcotic drugs and psychotropic substances, and Council Directive 92/109/EEC of 14 December 1992, on the manufacture and marketing of certain substances used in the illicit manufacture of narcotic drugs and psychotropic substances [17,18]. Each member state ensured that its Europol national unit and its representative in the European Information Network on Drugs and Drug Addiction (REITOX) network provided the EDU or the EMCDDA with information on the production, trafficking, and use of new synthetic drugs taking into account the respective mandates of these two organizations. The EDU and the EMCDDA would collect the information received, exchange it with each other, and forward it immediately, as appropriate, to the Europol national units, the representatives of the member states in the REITOX network, the Commission, and the EMA. This information had to include:

- a description of the chemicophysical characteristics and the name of the new synthetic drug;
- information on chemical precursors.

The article "New Psychoactive Substances: Evolution in the Exchange of Information and Innovative Legal Responses in the European Union" was published in 2020. Journal: Int J Environ Res Public Health.

At the request of any of the member states or the Commission, the EMCDDA was to convene, under the aegis of the Scientific Committee, a special meeting open to the experts nominated by the member states, to which representatives of the Commission, the EDU, and the EMA were invited. Once the risk assessment was completed, a report on the results would be drawn up, covering all aspects and giving all the opinions expressed. The risk assessment was to be carried out on the basis of the information provided by the member states, the Commission, the EMCDDA, the EDU, and the EMA, taking into account all the factors that, under the 1971 United Nations Convention on Psychotropic Substances, justified the decision to submit a substance to international control. On the basis of the proposed initiative, within one month of the date of the report on the results of the risk assessment, the Council could, on the basis of Article K.3(2)(b) of the Treaty, unanimously adopt a decision defining the new synthetic drug(s) to be made subject to the necessary measures or control. This framework allowed Europe to detect, assess, and respond to public health and social threats caused by the rapid spread of such substances.

### 3.3. Exchange of Information on New Synthetic Drugs (2005)

European Council Decision 2005/387/JHA of 10 May 2005 (Figure 1), on the information exchange, risk assessment, and control of NPS replaced the 1997 Joint Action (97/396/JHA) on new synthetic drugs [19]. This decision provided for an assessment of the risks posed by NPS so that control measures could be applied. The text was applied to the substances that were not listed in the tables of the 1961 United Nations Single Convention on Narcotic Drugs, but could pose a threat to public health similar to that of the substances listed in the tables and/or the 1971 United Nations Convention on Psychotropic Substances. Each EU country ensures that its Europol national unit and its representative to the REITOX provide information on the manufacture, trafficking, and use of NPS and preparations containing NPS. Europol and the EMCDDA collect the information transmitted by the EU countries using a reporting form and, in addition to communicating it to each other, immediately forward it to the Europol national units, the EU countries’ representatives within the REITOX, the European Commission, and the EMA. Therefore, in the light of the information transmitted by the EU member states, Europol and the Centre can submit where necessary a joint report including, inter alia, information on the involvement of criminal organizations in the manufacture or trafficking of an NPS, an initial indication of the risks posed by the substance itself, in particular, to health and society, as well as the characteristics of the users, the date on which the NPS was notified to one or other entity, etc. The EMA, in turn, informs Europol and the Center whether in the EU or in an EU country whether:

- the NPS had obtained a marketing authorization;
- the NPS was undergoing an authorization request;
- a marketing authorization granted for the NPS had been suspended.

The article "New Psychoactive Substances: Evolution in the Exchange of Information and Innovative Legal Responses in the European Union" was published in 2020. Journal: Int J Environ Res Public Health.

The Council, taking into account the opinion of Europol and the Centre, can request an assessment of the health and social risks arising from the consumption, production, and trafficking of an NPS, the involvement of criminal organizations, and the possible consequences of control measures. The risk assessment report specifies the psychochemical characteristics of the new substance, the health and social risks posed by its consumption, the chemical precursors used for manufacture, etc. No risk assessment is carried out in the absence of a joint report by Europol and the Centre, or if the assessment of the NPS is at an advanced stage of evaluation within the United Nations system, or if the Committee of Experts on Drug Addiction at the World Health Organization (WHO) has published its critical analysis accompanied by a written recommendation. No evaluation is conducted if the new substance has been used to manufacture a medicinal product already covered by an authorization or a suspended marketing authorization application. After receiving the risk assessment report, the Commission presents to the Council an initiative to submit the NPS to control measures. If the Commission does not consider it necessary to activate measures, these could be proposed to the Council by one or more EU countries. If the Council decides to submit an NPS to control measures, the EU countries endeavor to take the necessary steps to initiate control measures and to activate the criminal sanctions provided for in the legislation in accordance with their obligations under the 1971 UN Convention on Psychotropic Substances and the 1961 UN Single Convention on Narcotic Drugs. The Centre and Europol submit to the European Parliament, the Council, and the Commission an annual report on the effectiveness and results of the system implemented by the Decision. The EU countries and the EMA ensure the appropriate exchange of information between the mechanism established by the Decision and the pharmacovigilance systems established in accordance with Title VII of Directive 2001/82/EC and Title IX of Directive 2001/83/EC [20,21]. In 2006, the European Parliament and the Council of the European Union updated the regulation (EC Regulation No. 1920/2006) [22] of the EMCDDA created in 1993 (Regulation (EEC) 302/93 is repealed by Regulation (EC) 1920/2006) in order to provide concrete objective, reliable, and comparable information at the EU level on the “drug” phenomenon, on new psychoactive substances, on new ways of consumption (such as poly-drug use which combines the use of legal and illegal psychotropic drugs), on the consequences and risks, on the best practices and guidelines adopted in the member states, and on the results achieved. Therefore, the EWS system, which has existed since 1997, while keeping the three-step approach, has been revised and strengthened to cope with the increasing spread of new psychoactive substances. Moreover, the term “new psychoactive substances” was also used for the first time and given legal meaning, being defined as the substances not currently listed in any of the schedules to the United Nations Single Convention on Narcotic Drugs.

The article "New Psychoactive Substances: Evolution in the Exchange of Information and Innovative Legal Responses in the European Union" was published in 2020. Journal: Int J Environ Res Public Health.

### 3.4. National Laws and New Psychoactive Substances

Each country of the European Union could legislate on drugs with the national legislation in compliance with international conventions; therefore, measures to reduce both demand and supply of NPS began developing throughout Europe. Individual member states have taken steps to improve and accelerate legal responses to these new substances, their products, and the structures that marketed them. While most European countries have continued to update the list, many have responded with innovative changes to their legislation or enforcement policies. At the national level, various measures have been taken to control new substances. Three general types of legal strategies were identified:

- existing laws regarding issues unrelated to controlled drugs are used, such as consumer safety legislation;
- existing drug laws or procedures are expanded or adapted;
- new legislation is developed.

#### 3.4.1. Countries Using Consumer Safety or Medicines Legislation

A number of European countries have successfully stopped the distribution of NPS using the existing legislation with little changes.

Consumer safety or medicines laws based on the harmonized European Union (EU) definitions have been operative in all the European states. The consumer protection laws have been adopted in different countries: some of these were targeted towards psychoactive products in general, as in Poland, where there has been a mass closure of “headshops”, whereas the other ones faced single substances [23]. In Italy, for example, the regulations for the correct identification and packaging of goods and food have been used to seize herbal products that contained synthetic cannabinoids that are not labelled in Italian. A similar strategy was used in the United Kingdom to prevent mephedrone sale as bath salts or plant-based products. Later, Poland changed the definition of a “substitute drug”, initially meaning a substitute of a drug or a substance with similar uses, and reinforced its health protection law to use it if a substitute drug is suspected to be the cause of health harms. The European definition of a medicinal product that does not require that the product has healing properties has allowed the use of this regulation to hinder the spread of new psychoactive substances. In this way, if an NPS had been classified as a medicinal product, the national medicines agency could have required an authorization for its importation, supply, or sale: eight countries used these laws to control the distribution of NPS. Notwithstanding, in July 2014, the Court of Justice of the European Union ruled that substances are not medicinal products if they do not have beneficial effects on human health, thus restricting the use of such laws for NPS control and making this approach no more practicable [24].

The article "New Psychoactive Substances: Evolution in the Exchange of Information and Innovative Legal Responses in the European Union" was published in 2020. Journal: Int J Environ Res Public Health.

#### 3.4.2. Modification or Extension Of Existing Laws

For several European countries, an alternative response to the threat of NPS was their managing by modifying or extending the preexisting drug legislation. In Hungary (2010) and Finland (2011), for example, scientific committees were constituted to provide for the lack of information on new drugs and to contribute to their control with science-based evidence decisions [25]. In several countries, temporary controls were introduced to facilitate and hasten legal processes: these procedures were legislated and enforced in Latvia and Slovakia in 2013 by the Center for Disease Prevention and Control and the Minister of Health, respectively. Similar approaches to add non-therapeutic substances to the lists of the controlled drugs were enacted in the United Kingdom and in Hungary in 2011 and 2012, respectively, authorizing, for example, temporary orders of specific classes of drugs to control them as scheduled substances under drug regulation. To stem the wide spread of these new substances, the administrative offence for personal possession was introduced in 2014 in Latvia, whereas possession of more than 10 g of an active substance was outlawed in Hungary. In 2014, in the Czech Republic, a parliamentary law followed by new government decrees was promulgated to list the controlled drugs and limit the time for scheduling. In the same year, in Finland, the Narcotics Act was extended to include prohibited psychoactive substances and extend the offence against public health and safety to this threat with sentences up to a year of prison for the offenders. Some countries extended their preexisting drug regulation to well-defined groups of substances in place of single compounds, such as Luxembourg, Italy, Cyprus, Lithuania, Denmark, France, Norway, Croatia, and Turkey. In Finland, the definition of “positional isomers for such a substance” was introduced in the drug laws and Germany adopted the “group definition” approach: conversely, in 2012, the Netherlands refused these innovative strategies because of the difficulties of targeting some compounds which might have had useful applications in the pharmacological field [26].

The article "New Psychoactive Substances: Evolution in the Exchange of Information and Innovative Legal Responses in the European Union" was published in 2020. Journal: Int J Environ Res Public Health.

#### 3.4.3. Developing New Regulations to Hinder Spread of New Substances

In most of the EU countries, new legislations have been enacted to counter the illegal distribution of new drugs, e.g., in Ireland, Austria, Portugal, Romania, Sweden, and the United Kingdom. Despite common purposes, several differences can be evidenced in the development of the legislation between these countries. Except Sweden, the other states have defined a psychoactive substance as a compound that is a stimulant or a depressor of the central nervous system; in Ireland, Austria, Portugal, and Romania, this definition is also related to a condition of dependence, onset of hallucinations, and behavioral or motor functional disturbances, whereas in the United Kingdom, the term “psychoactive” is closely related to a condition of alteration of the person’s mental or emotional state. These disorders have to be “relevant” in Ireland and Portugal to lead to a new drug law, whereas in Austria, these substances are included in a list only if they are recognized as compounds potentially able to cause addiction. In Romania and in the United Kingdom, instead, there is no need to demonstrate the real health harm of these new substances. As a consequence of the new regulation, in Ireland, Romania, and the United Kingdom, all the substances with the characteristics stated in the law are enclosed in it without being explicitly mentioned in the legislation. Conversely, in Austria, the substances have to necessarily be named according to the dispositions of the Minister of Health. In Portugal, although the drugs are reported in an Administrative Rule, the government has the ability to seize and analyze all the substances suspected to be dangerous for the public health, forbidding their sale. Furthermore, the distribution of psychoactive substances in Austria is an offence if the supplier is aware of their effects; in the United Kingdom, the dealer has to be informed about the purposes of the purchase, whereas in Ireland, it is mandatory to indicate if the goods are likely for human consumption. In Romania, none of these dispositions are necessary. In Ireland, Romania, and the United Kingdom, the maximum penalty for the distribution of the psychoactive substances is respectively five, three, and seven years of imprisonment. In Austria, two years of imprisonment are sanctioned for the same offence with an increase of the penalty in the event of health harm or death. Promoting the sales of these drugs is punished with five years of prison in Ireland, from one to three years in Romania, and up to eight years in the Czech Republic in case of advertising of the addiction to an NPS. In Romania, the “legal” sales of these compounds is punished with three to ten years of prison and big penalties have been established for not removing specific websites upon request of the Ministry. In Poland, heavy fines are imposed in case of substitute drug supply and the promotion of such substances is condemned with one year of prison. The law innovation is a continuously evolving process. Since 2009, seven countries have implemented their own regulatory system: in Portugal, only administrative fines have been established for these crimes and the opportunity for closing shops selling NPS has been given to the authorities. In Sweden, in 2011, administrative power for seizing dangerous substances was entrusted to police forces and customs. Despite the numerous differences in regulatory approaches to the problem of NPS in Europe, two common lines of work can be outlined: the risk of imprisonment for traffickers with severe penalties and heavy fines for personal use of drugs [25]. At the national level, a number of measures have therefore been taken to control new substances using three different types of legal response. In some countries, existing laws relating to the issues unrelated to controlled drugs have been used, such as legislation on consumer safety; in others, existing laws or procedures on drugs have been expanded or adapted; in others, new legislation has been developed. Although a wide range of offences and sanctions have been defined for all countries, responses have often focused on measures to prevent supply rather than possession of these substances.

The article "New Psychoactive Substances: Evolution in the Exchange of Information and Innovative Legal Responses in the European Union" was published in 2020. Journal: Int J Environ Res Public Health.

### 3.5. National Risk Assessment Procedures

In 2008, the EMCDDA carried out a study on the different national legal procedures involved in bringing new substances under the control of drug legislation, the time required by this procedure, and if national risk assessment procedures were involved. Three different approaches to risk assessment emerged in the 26 countries examined. These systems examined the social and health risks posed by these substances at different stages from production to trafficking and use. They could also assess the potential involvement of organized crime and the consequences of possible control measures. In six countries, no national risk assessment was carried out (Belgium, Ireland, Greece, Spain, Hungary, Finland) [26]. These countries were generally relying on risk assessments carried out at the international or the European level. In seven countries, national risk assessments could be carried out only if necessary (Czech Republic, Cyprus, Latvia, Luxembourg, Poland, Portugal, Slovenia) [26]. In 13 countries, a type of risk assessment was carried out to consider whether to control a substance as required by a drug law or equivalent text or as part of the procedure required to propose new legislation (Denmark, Germany, Estonia, France, Lithuania, Netherlands, Austria, Romania, Sweden, the United Kingdom, Croatia, Norway, Slovakia) [26]. The damage levels found did not affect the speed of the legislative process in 12 of the 20 countries. Four countries (Germany, Luxembourg, Slovakia, Sweden) could switch to a shortened legislative procedure if risk levels were considered high. In France, Austria, and Norway, cases of urgency led to a shortened duration of the risk assessment itself. In the Netherlands, both options were available. In 16 countries, national risk assessments were carried out by a group of experts within the public administration, which could be a competent ministry or a state or government agency. Six countries provided or could provide the opportunity to consult independent scientists if the need was perceived. In three countries (Netherlands, Austria, United Kingdom), risk assessment was carried out by independent scientific organizations. Approximately half of the EU member states legally distinguished substances according to their harmfulness; risk assessment could contribute to this by providing precise classifications and information on harm to the public. Risk assessment was therefore a process aimed at identifying, analyzing, and quantifying the health risks (including potential ones) but also the social and criminal risks associated with NPS intake.

The article "New Psychoactive Substances: Evolution in the Exchange of Information and Innovative Legal Responses in the European Union" was published in 2020. Journal: Int J Environ Res Public Health.

### 3.6. Exchange of Information on New Synthetic Drugs (2013)

In 2011, following a review of the system, the European Commission considered a new instrument to replace Council Decision 2005/387/JHA. Under the current EU instrument, Council Decision 2005/387/JHA, the Commission could propose to the member states to make new drugs subject to criminal law measures. This mechanism allowed 9 substances to be made subject to restriction measures and criminal penalties. Recently, in 2010, the Commission proposed and obtained an EU-wide ban on mephedrone, a drug similar to ecstasy (MEMO/10/646), and, in early 2013, on the substance 4-methylamphetamine (4-MA), similar to amphetamine (IP/13/75). In June 2013, the Commission also proposed to ban the synthetic drug 5-(2-aminopropyl)indole (5-IT) (IP/13/604). A 2011 report showed that the current system was struggling to keep pace with the large number of new substances appearing in the market. The procedure for submitting a single substance to restrictive measures took two years. Criminals could then circumvent the control measures by making minor changes to the chemical structure of the substance without mitigating its serious health consequences. In addition, the binary nature of the current system (with only two options: criminal measures or no action) hampered the European Union’s ability to act by not allowing it to consider effective options for rapid and targeted control measures. The Commission’s assessment of the functioning of Council Decision 2005/387/JHA on NPS concluded that the Decision had three main shortcomings: it was unable to cope with the sharp increase in the number of NPS, and this was because it only dealt with one at a time, with a time-consuming procedure; the substances subject to control measures were quickly replaced by new substances with similar effects; it did not provide sufficient options for regulatory and control measures. Therefore, on 17 September, 2013, the European Commission proposed to make NPS illegal according to a new procedure that aimed to update the one previously reported in European Council Decision 2005/387/JHA, making it faster and more effective (IP/11/1236). The proposal stemmed from proposals by the European Medicines Agency and the European Observatory to strengthen the current European mechanisms for tackling NPS. The new system was based on a totally different approach. Substances posing a moderate risk were permanently restricted to the consumer market, while those posing a high risk were completely restricted. Only the most harmful substances, which led to a serious risk to consumer health, were subject to criminal measures. With such an instrument, European action to identify, assess, and withdraw NPS from the market could become much faster:

- In case NPS represented an immediate risk, measures could be introduced throughout the EU within a few weeks, for a period of one year, to restrict their sale to consumers (temporary measures).
- In the case of a serious risk, permanent measures could be introduced within 10 months (compared to the previous two years), which not only limited the sale of NPS, but also restricted their use in the industrial sector (permanent measures).

The article "New Psychoactive Substances: Evolution in the Exchange of Information and Innovative Legal Responses in the European Union" was published in 2020. Journal: Int J Environ Res Public Health.

Specifically, in the event that an NPS raised concerns at the European level about the health, social, and security risks it might entail, the European Observatory and Europol would draw up a joint report on the substance. On the basis of this report, the Commission would decide whether there were grounds for requiring a proper risk assessment. If the Joint Report showed that the substance posed immediate risks to public health (e.g., it was highly toxic and caused fatal accidents across Europe), the Commission would also place it under a temporary restriction in the market. This prevented the sale of the substance for one year, but its legitimate uses were not affected by the measure. In this way, consumers were considered to be protected during the risk assessment of the substance, while industrial, commercial, or scientific uses were not hindered. No action was taken if the substance involved low risks (low); banning the substance to the consumer market if the risk was moderate (moderate); banning the substance from the consumer market and restricting its commercial and industrial uses if it presented serious (severe) risks. In addition, there are also criminal measures. Within one year, member states had to act to make the substance subject to the criminal provisions applicable to drugs, including at the national level. Unlike the current system, the new measures were directly applicable in the member states and did not need to be transposed into a national law (MEMO/13/790). This allowed the EU’s response to harmful NPS to be significantly accelerated. Moreover, under the new mechanism, the European Monitoring Centre could also include in its evaluation the substances similar to the one already formally under consideration. This was in order to anticipate the marketing of new substances by criminals who tried to circumvent the restrictive measures by making minor changes to the chemical structure of a banned substance. Therefore, the European Commission proposed to make NPS illegal according to a new procedure that aimed to update the one previously set out in European Council Decision 2005/387/JHA, making it faster and more effective (IP/11/1236) (Figure 2). The proposal stemmed from the proposals of the EMCDDA and the need to strengthen the existing European mechanisms to tackle NPS. The new system would allow an approach where substances posing a moderate risk would be permanently restricted to the consumer market, while those posing a high risk would be completely restricted. Only the most harmful substances, which pose a serious risk to consumer health, would be subject to criminal measures.

The article "New Psychoactive Substances: Evolution in the Exchange of Information and Innovative Legal Responses in the European Union" was published in 2020. Journal: Int J Environ Res Public Health.

### 3.7. Exchange of Information on New Synthetic Drugs (2018)

In 2017, 51 NPS were reported for the first time to the EU EWS, averaging one substance per week [27]. At the end of 2017, the Centre reported that it was tracking 670 new psychoactive substances (compared to 350 in 2013) [27]. Social and health problems related to new synthetic cannabinoids and opioids (mainly intoxications and deaths) prompted the agency to conduct nine new risk assessments in 2017, an unprecedented amount. Across Europe, since 23 November 2018, the EU EWS and risk assessment procedures for NPS have been strengthened and control processes—accelerated (Regulation (EC) No. 1920/2006 is amended by Regulation (EU) 2017/2101). Legislation had to keep pace with the recent growth in these substances and new proposals from the European Commission (EC) followed. This new legislative framework included:

- a regulation for the exchange of information, an early warning system, and a risk assessment procedure for new psychoactive substances amending the existing Regulation in the EMCDDA (European Monitoring Centre for Drugs and Drug Addiction);
- a directive allowing NPS to be controlled at the EU level as “drugs.”

The legislation retained the current European three-step approach to react to NPS (early warning, risk assessment, and control measures), considerably strengthening the existing procedures by streamlining and accelerating data collection and evaluation procedures. A new feature of the Regulation made it possible to jointly assess the potential risks posed by several NPS with a similar chemical structure through a single risk assessment report. Shorter deadlines applied to all these new procedures. The EMCDDA continued to play a leading role in alerting and observing NPS reported by EU member states and it became its task to launch an in-depth scientific study on all new substances of concern at the EU level. After the Agency has submitted its initial report, the European Commission will have two weeks to ask the EMCDDA itself to assess the potential risks posed by the substance. This evaluation will have to be remitted within six weeks. Based on the risk assessment report, the Commission may propose to control the substance. The Council of the EU and the European Parliament will then have two months to accept or not accept these proposals. Authorities of the member states will have six months (instead of 12 months under the old system) to put the substance under national control once the decision comes into force. Under the new legislation, other EU agencies will be involved, including the ECDC, the ECHA, and the EFSA. Finally, the European Commission amended the annex of Council Framework Decision 2004/757/JHA by including NPS in the definition of “drugs” with Commission Delegated Directive (EU) 2019/369 of 13 December 2018 [27]. The new legislative framework that has been applied since November 2018 has been offered to the European Union as a major tool in helping achieve major protection of the health and security of people living in Europe (Figure 3).

The article "New Psychoactive Substances: Evolution in the Exchange of Information and Innovative Legal Responses in the European Union" was published in 2020. Journal: Int J Environ Res Public Health.

## 4. Discussion

The worldwide phenomenon of NPS has always represented a challenging issue due to its changing nature. The continued availability of NPS has increased the complexity of the drug phenomenon in Europe. The range of substances and products has grown, as well as the number of consumers for recreational use, self-medication, stimulating purposes, or problematic use. The phenomenon also revealed the interactions between the markets for new substances and illicit drugs, because new substances are increasingly being sold directly into the illegal market and passed off as illicit drugs when, for example, they are missing from the market. This indicates that in the global context, Europe is an important market for drugs, supported by both domestic production and illicit imports of drugs from other regions. Latin America, West Asia, and North Africa are important supply areas for the drugs arriving in Europe, as well as for some drugs and precursors transiting from Europe to other continents. In this concern, the European system has been revised at both the national and the central level with the aim of establishing a faster and more effective system. The new legislation, while maintaining the three-step approach—early warning, risk assessment and control measures—has strengthened the existing processes, streamlining and accelerating data collection and evaluation procedures and introducing shorter deadlines. In response to the risk evaluation proposed by the EMCDDA, the Council promulges decisions which are transposed by the member states according to their legislation system. The changes also strengthen the network supporting the EMCDDA and Europol in this work, with formal working arrangements between the EMCDDA and the EMA, the EFSA, the ECDC, and the ECHA. Anyway, it should be considered that the current legislation is not yet effective in preventing the emerging NPS spread and the evolution of the phenomenon. For decades, the three United Nations drug conventions have served as the basis for member states’ obligations and international cooperation on drug control, but there is no international consensus on legislative control of NPS. The emergence of new psychoactive substances (NPS) poses a new global public health risk and a challenge to global drug policy, as there is a lack of international consensus on the legislative control of NPS. In summary, the different legislative approaches used can influence the results of NPS control. For example, Taiwan, S. Korea, and Japan adopted a similar attitude toward the management of controlled drugs, but the legislative criteria and the procedure for NPS scheduling/listing are quite different [28]. Japan’s approach covers the gray area between legal pharmaceuticals and illegal drugs. The legislative approaches in S. Korea and Japan allow timely monitoring of NPS, prompt implementation of declaring NPS illegal drugs, and systematic regulation of NPS. In Taiwan, NPS are listed as controlled drugs only when they are identified to possess addictive potential, illicit use liability, and social harm liability. These rigid criteria explain, at least in part, why there are only few NPS controlled in Taiwan. In the United States, the Controlled Substances Act (CSA) contains the federal drug policy, under which the manufacture, importation, possession, use, and distribution of certain substances is regulated. For the purposes of control, the CSA places all substances into one of five schedules based upon the substance’s medicinal value, harmfulness, and potential for abuse or dependence. Temporary scheduling of new substances to avoid imminent hazard to public safety is also possible under the CSA. In 2011, several synthetic cannabinoids (JWH-018; JWH-073; JWH-200; CP-47,497; CP-47,497 C8 homologue) [29] and some synthetic cathinones (mephedrone; methylone; and 3,4-methylenedioxypyrovalerone (MDPV)) [30] were subject to temporary control. In addition to the CSA, the United States has a Controlled Substances Analogue Enforcement Act, i.e., the “Federal Analogue Act”, to control substances not specifically listed in the CSA. The enactment of the Federal Analogue Act in 1986 was a response to the spread of fentanyl derivatives, α-prodine derivatives, phenethylamines related to MDMA, amphetamines, and other compounds designed to produce effects similar to the controlled drugs they mimic. Due to the absence of a global early warning system which monitors the appearance of new substances, the United Nations Office on Drugs and Crime (UNODC) thus developed the first international monitoring system on new psychoactive substances (NPS) under the Global Synthetics Monitoring: Analyses, Reporting and Trends (SMART) Programme [31]. The UNODC Early Warning Advisory (EWA) on new psychoactive substances (NPS) was established in 2013 following a resolution passed by the member states at the Commission on Narcotic Drugs as a response to the emergence of NPS at the global level. The EWA serves as a tool for effective, evidence-based policy responses by monitoring, analyzing, and reporting global and regional trends on NPS. The EWA thus serves as a repository for information on NPS leading to an improved understanding of their distribution and use at the global level and offers a platform for the provision of technical assistance to the member states. The EWA has enhanced its features by including toxicology data in order to identify the NPS which pose the greatest threat to public health, thus assisting in the prioritization of the substances assessed for international control as well as legislative responses at the national level. The reporting countries arise from geographical regions which include North America, Europe, Asia, and Oceania. Although the analysis allows for a broader understanding of the associated harm of NPS, it is not an exhaustive representation of the variety and toxicity of NPS present globally. 

The article "New Psychoactive Substances: Evolution in the Exchange of Information and Innovative Legal Responses in the European Union" was published in 2020. Journal: Int J Environ Res Public Health.

## 5. Conclusions

Apart from possible wider effects on policies on new psychoactive substances, the existence of a global market for these substances stimulates innovation and the development of new products, encourages research and distribution of uncontrolled substitutes that could, over time, change consumption patterns in Europe. In this respect, the existence of a worldwide monitoring system to assess potential health implications and to implement timely and targeted worldwide responses by legislators and law enforcement authorities is essential.

## Figures and Tables

**Figure 1:** Procedure applied according to the European Council Decision 2005/387/JHA.

**Figure 2:** New procedure according to IP/11/1236.

**Figure 3:** Shorter deadlines of the New Release No. 8/2018 procedure compared to the European Council Decision 2005/387/JHA procedure. The illustration is a simplified version of the figure available in the EMCDDA page at https://www.emcdda.europa.eu/publications/topic-overviews/eu-early-warning-system.
